# Short-Term Efficacy and Quality of Life of Gastric Cancer Patients Undergoing Radical Gastrectomy Assisted by External Vision

This article has been retracted.

**DOI:** 10.1155/2021/4256347

**Published:** 2021-12-02

**Authors:** Jian Zheng, Yingwei Xue, Chunfeng Li

**Affiliations:** ^1^Department of Diagnostic Radiology Division, Harbin Medical University Cancer Hospital, Harbin 150081, China; ^2^Department of Gastrointestinal Surgical Ward, Harbin Medical University Cancer Hospital, Harbin 150081, China

## Abstract

**Objective:**

To evaluate the clinical effects and survival prognosis of radical gastrectomy assisted by external vision in gastric cancer.

**Methods:**

A total of 60 hospitalized gastric cancer patients from June 2016 to December 2018 were selected and divided into the observation group and control group according to different surgical procedures. The control group was treated with traditional open radical gastrectomy, while the observation group was treated with radical gastrectomy assisted by an external vision microscope. Relevant surgical indicators, visual analogue scale (VAS), postoperative complications, and life quality assessment were analyzed and compared between the two groups.

**Results:**

The incision length and intraoperative blood loss in the observation group were smaller than those in the control group, and the difference was statistically significant (*P* < 0.05); compared with the control group, the observation group had significantly shorter hospital stay, earlier postoperative first exhaust time, and lower gastric fluid volume at the 3^rd^ day after surgery (*P* < 0.05). The pain scores of the observation group at 1, 4, and 12 weeks after surgery were lower than those of the control group (*P* < 0.05), and the difference was significant. The quality of life scores at the 1^st^ week and 12^th^ week after surgery showed that the dysphagia symptom scores of the observation group and the control group were significantly reduced but the two groups had significant differences in fatigue, physical function, pain score, postoperative pain, and overall quality of life. The observation group was significantly better than the control group (*P* < 0.05). Follow-up studies showed no significant difference between mortality and cancer recurrence (*P* > 0.05); the patients recovered well at postoperation, and the diet of the observation group was better than that of the control group (*P* < 0.05); gastric reflux and knife pain were less than those of the control group (*P* < 0.05).

**Conclusion:**

Radical gastrectomy assisted by external vision for gastric cancer yields clinical benefits for gastric cancer patients, which not only dramatically shortened the length of hospital stay but also effectively ameliorated the quality of life of patients, all indicating that external vision-assisted surgery was significantly better than traditional gastrectomy in improving the postoperative quality of life of gastric cancer patients in the absence of increasing the risk of adverse events.

## 1. Introduction

Gastric cancer is one of the widely occurred malignant neoplasms. As the latest data revealed that the incidence and mortality of gastric cancer rank 6^th^ and 3^rd^ worldwide, respectively [1], and that in China, they are rank 2^nd^ and 3^rd^, respectively [2]. At present, surgical treatment is a common method for gastric cancer. The survival time can be effectively prolonged through resecting neoplasms or by other treatments. Traditional open surgery brought about great trauma to patients and it is not conducive to postoperative recovery [3]. However, laparoscopic surgery has been gradually applied in the treatment of a variety of abdominal diseases, which has the characteristics of less trauma, fewer complications, quick postoperative recovery, good clinical effect and so on but also has certain risks. With the development of technology, the auxiliary technology of external vision mirror has been gradually applied in the clinic. The purpose of this study was to investigate the clinical effects and prognosis of patients with gastric cancer who underwent radical gastrectomy assisted by a laparoscope and radical gastrectomy assisted by laparotomy.

## 2. Materials and Methods

### 2.1. Research Objects

A total of 60 patients with gastric cancer admitted to our hospital from June 2016 to December 2018 were collected and divided into the observation group (24 cases) and control group (36 cases) according to the surgical method. Inclusion criteria are as follows: (1) the patient was diagnosed as gastric cancer by examination and received surgical treatment for the first time, (2) the patient has no serious diseases of the blood system or other organs, and (3) patients volunteered to participate in this study. Exclusion criteria are as follows: (1) patients with severe chronic wasting disease, hypertension, cardiopulmonary failure, and other diseases and surgical contraindications, (2) a history of surgical treatment of the stomach and abdomen, and (3) other malignant tumors or other autoimmune diseases. There were no statistically significant differences in gender, age, tumor diameter, or TNM stage between the two groups (*P* > 0.05). The data were comparable, as shown in Table 1.

### 2.2. Surgical Methods

#### 2.2.1. Observation Group

Endotracheal intubation combined with intravenous anesthesia was performed in the supine position. The Vitom2/3D optometry surgical system with HD video assistance was adopted in the middle of the upper abdomen (7–9 cm). Depending on the site of the tumor, the surgical procedure (radical total or distal subtotal gastrectomy) was performed.

#### 2.2.2. Control Group

General anesthesia was performed with tracheal intubation. The incision was made around the umbilicus at 20–30 cm in the middle of the upper abdomen. Traditional D2 radical gastrectomy was performed.

### 2.3. Observation Index

(1) The hospitalization time, operation time, incision length, intraoperative blood loss, number of lymph node dissection, postoperative first exhaust time, postoperative gastric juice volume, gastric tube extubation time, eating time, and so on were statistically compared between the two groups. (2) The pain visual analogue score was used to score the pain degree of the two groups at 1 week, 4 weeks, and 12 weeks [4]. The smaller the value was, the lighter the pain was. After treatment, the subjective score of the same period of time was recorded according to the degree of pain felt by the patients and the average value was compared. (3) The Chinese versions of EORTC QLQ-STO22 and EORTC QLQ-30 were used to evaluate the quality of life [5, 6]. The EORTCQ LQ-C30 (version3.0) score was obtained from the patient's self-evaluation, which included five functional indexes: role function, cognitive function, physical function, social function, emotional function, vomiting or nausea, pain, and fatigue, as well as 30 other items. EORTC QLQ-STO22 was a special module for patients with gastric cancer, including 9 subscales and 22 items: gastric cancer patients have specific symptoms: a total of 22 items such as body appearance, hiccups, dysphagia, stomach pain, and dysphagia. The follow-up study was conducted within 1 week before operation and 1 week and 12 weeks after operation. The higher the EORTC QLQ-30 functional index dimension score and the comprehensive quality of life dimension, the higher the quality of life; the lower the EORTC QLQ-STO22 symptomatic index dimension and the EORTC QLQ-STO22 gastric cancer-specific symptom score, the lighter the symptom and the better the quality of life.

### 2.4. Statistical Analysis

SPSS 21.0 software was used for statistical analysis. The quantitative data were represented by ($\bar{x}\pm s$). The *χ*^2^ test was used for comparison of count data. The *t*-test was used for comparison between groups and the Mann–Whitney *U* nonparametric test for nonnormal distribution data (*P* < 0.05).

## 3. Results

### 3.1. Comparison of Intraoperative Clinical Efficacy between the Two Groups

The incision length and intraoperative blood loss in the observation group were smaller than those in the control group, and the difference was statistically significant (*P* < 0.05). Although the operation time of the observation group was less than that of the control group and the number of lymph node dissection was more than that of the control group, the difference was not significant (*P* > 0.05), as shown in Table 2.

### 3.2. Comparison of Postoperative Clinical Efficacy Indexes between the Two Groups

Compared with the control group, patients in the observation group had significantly shorter hospital stay, significantly earlier postoperative first exhaust time, and lower gastric fluid volume on the third day after surgery (*P* < 0.05). There was no statistically significant difference between the two groups in gastric tube removal time and eating time (*P* > 0.05), as shown in Table 3.

### 3.3. Comparison of Pain Visual Simulation Scores between the Two Groups (VAS)

The pain scores of the study group at 1, 4, and 12 weeks after surgery were lower than those of the control group (*P* < 0.05), and the difference was significant, as shown in Table 4.

### 3.4. EORTC QLQ-30 and EORTC QLQ-STO22 Were Used to Compare Patients' Quality of Life

Data of 1 week before surgery showed that there was no statistical difference between the two groups in terms of preoperative functional dimension and symptom dimension (*P* > 0.05), indicating comparability. The quality of life scores at the 1st week and 12th week after surgery showed that the dysphagia symptom scores of the observation group and the control group were significantly reduced but the two groups had significant differences in fatigue, physical function, pain score, postoperative pain, and overall quality of life. The observation group was significantly better than the control group (*P* < 0.05). There were no significant differences in other general indicators of EORTC QLQ-30 or in the specific quality of life dimensions of EORTC QLQ-STO22 and other gastric cancer patients (*P* > 0.05), as shown in Table 5.

### 3.5. Postoperative Follow-Up of Two Groups of Patients

As shown in Table 6, there was no significant difference between patient death and cancer recurrence and metastasis (*P* > 0.05). The patients recovered well after operation, and the diet of the observation group was better than that of the control group (*P* < 0.05); gastric reflux and knife pain were less than those of the control group (*P* < 0.05).

## 4. Discussion

Gastric cancer is a malignant tumor originating from gastric mucosal epithelium and usually occurred at the age of 50 years. Nevertheless, because of the pressure of work, diet changes, and *Helicobacter pylor*i infection, the incidence rate of gastric cancer in China has been younger and younger. At present, the main treatment of gastric cancer is surgical resection combined with radiotherapy and chemotherapy; the most important part of which is radical gastrectomy (D2) [7, 8]. In 1991, Goh et al. reported the first laparoscopic-assisted distal gastrectomy, and in 1997, Goh et al. reported laparoscopic-assisted radical gastrectomy (D2) for advanced gastric cancer. After >10 years of development, laparoscopic surgery of gastric cancer is becoming increasingly diverse, surpassing the common type of traditional surgery [9, 10]. Although laparoscopy has many advantages, it also has some limitations. For example, studies have shown that laparoscopic-assisted radical gastrectomy for gastric cancer takes a long time to operate. Another example is the difference in lymph node dissection due to the uneven technique of the surgeon, which affects the prognosis. In addition, laparoscopic technology is limited by the patients' physical conditions, such as their advanced age, poor cardiopulmonary function, and especially chronic lung diseases, which make the patients have poor tolerance to carbon dioxide pneumoperitoneum.

With the development of medical technology, the external vision auxiliary system can make the surgical field of vision clearer, greatly improve the success rate of surgery, and shorten the operation time through 2D/3D transformation. There are no such disadvantages in minimally invasive surgery for gastric cancer assisted by external vision microscopy. The application of the far-infrared light (NIR/ICG) system and fluorescent contrast dye indocyanine green (ICG) can obtain real-time vision of the lymphatic system around the gastric cancer site under nonradiation conditions, which is very simple to operate. External vision mirror is an innovative medical device in the development of minimally invasive surgery. Different from the traditional endoscope, the external vision mirror is a “external vision mirror” placed 25–75 cm from the operating table. It is fixed by a supporting and fixation system to ensure that the doctor has enough operating space. With its flexible viewing angle and magnification function, the minimally invasive surgery for gastric cancer assisted by external vision mirror presents the operative images on the video display and the magnification of the tissue structure improves the accuracy of the surgery and ensures the correct diagnosis. At the same time, it enables doctors and medical staff to work clearly, comfortably, and harmoniously, greatly reducing doctors' sense of fatigue and saving time and effort. The autologous imaging system of the opticoscope has brought high-quality and ergonomic innovations to the view of open surgery.

The postoperative pain of patients undergoing surgery with optometrix had little effect on postoperative quality of life. At the same time, small scars after small incision do not affect the appearance and the postoperative recovery time is shorter [11]. In this study, the pain scores of the study group at weeks 1, 4, and 12 after surgery were all lower than those of the control group (*P* < 0.05), indicating that the incision pain and healing effect under the aid of an external vision microscope were significantly superior.

The present study compared the efficacy of radical gastrectomy assisted by laparoscopy and conventional open gastrectomy in the treatment of gastric cancer. The results showed that the incision length, intraoperative blood loss, length of hospital stay, first postoperative exhaust time, and gastric juice volume on the third day were significantly better in the observation group (*P* < 0.05), which was consistent with the research results [9, 10]. Follow-up results showed that the diet of patients undergoing radical gastrectomy assisted by an external vision microscope was better than that of the control group and gastric acid reflux and knife edge pain were less than those of the control group (*P* < 0.05). There were no significant differences in mortality and cancer recurrence rates between the two groups (*P* > 0.05). This result suggested that patients undergoing radical gastrectomy assisted by external vision have a better prognosis, which was conducive to patients' recovery, and there was no difference in mortality and recurrence rate compared with traditional surgery. Although there was no significant difference between the operation time of the observation group and the control group, the operation time of the control group was relatively short, indicating that the endoscopic assist system combined with a laparoscope shortened the operation time. And this may be attributed to its wide field of vision, clear imaging function, and more effective observation of the lesion area, so as to ensure a good surgical effect.

At present, it is more and more accepted in foreign countries to evaluate the quality of life through scale survey of patients' own feelings. As the first developed EORTC QLQ-STO22 and QLQ-C30 life quality evaluation systems, EORTC QLQ-STO22 and QLQ-C30 have been widely used in overseas studies on the quality of life of gastric cancer patients. Previous studies have shown that the quality of life of gastric cancer patients undergoing palliative care through EORTC QLQ C30, regardless of the overall health, physical, social function, and emotional aspects of the patients, is significantly better than that of the control group. Therefore, patients with gastric cancer who are eligible for surgery should undergo surgery [12–14]. However, comparative studies on the quality of life between different gastric cancer resections have been rarely reported. The quality of life scores at the 1^st^ week and 12^th^ week after surgery showed that the dysphagia symptom scores of the observation group and the control group were significantly reduced but the two groups had significant differences in fatigue, physical function, pain score, postoperative pain, and overall quality of life. The observation group was significantly better than the control group (*P* < 0.05). According to the data of this study, EORTC QLQ-C30 and EORTC QLQ-STO22. This study shows that the combined use of laparoscopic radical gastrectomy with external vision can increasingly shorten the duration of surgery and decrease the amount of intraoperative blood loss, which probably resulted from the improvement of surgeon's proficiency as well as the improvement of teamwork. Laparoscopic radical gastrectomy assisted by external vision is safe and feasible and superior to traditional surgery in the aspects of intraoperative blood loss, postoperative exhaust time, and postoperative hospital stay. Due to the limitations of our study, further larger and multicenter studies are needed to validate our findings.

## 5. Conclusion

In summary, radical gastrectomy assisted by external vision for gastric cancer yields clinical benefits for gastric cancer patients, which not only dramatically shortened the length of hospital stay but also effectively ameliorated the quality of life of patients, all indicating that external vision-assisted surgery was significantly better than traditional gastrectomy in improving the postoperative quality of life of gastric cancer patients in the absence of increasing the risk of adverse events.

## Figures and Tables

**Table 1:** The general information.

Group	*n*	Gender		Age	Tumor diameter		TNM staging	
		Male	Female		≤5 cm	>5 cm	I–II	III–IV
Control group	36	24	12	61.75 ± 9.33	22	14	33	3
Observation group	24	15	9	57.88 ± 9.51	19	5	22	2
*χ* ^2^/*t*		0.110		1.562	2.169		0.227	
*P*		0.740		0.124	0.141		0.634	

**Table 2:** Comparison of intraoperative clinical efficacy between the two groups.

Group	*n*	Operation time (min)	Incision length (cm)	Intraoperative blood loss (ml)	Lymph node dissection (n)
Control group	36	194.16 ± 31.72	8.47 ± 2.45	178.06, IQR (85, 275)	16.69 ± 2.17
Observation group	24	183.33 ± 34.48	6.98 ± 1.23	91.667, IQR (50, 100)	18.15 ± 3.82
*χ* ^2^/*t*/*Z*		1.251	2.752	−2.800	1.886
*P*		0.216	0.008	0.005	0.064

**Table 3:** Comparison of postoperative clinical efficacy indexes between the two groups.

Group	n	Hospital stay (d)	Postoperative first exhaust time (d)	Gastric fluid volume on the third day (ml)	Gastric tube removal time (d)	Eating time (d)
Control group	36	13.53 ± 5.27	5.194 ± 0.577	62.22, IQR (32.5, 60)	5.19 ± 0.58	5.58 ± 1.23
Observation group	24	10.38 ± 1.81	4.833 ± 0.565	35, IQR (20, 50)	4.88 ± 0.85	5.25 ± 0.68
*χ* ^2^/*t*/*Z*		2.814	2.396	−2.962	1.736	1.211
*P*		0.007	0.002	0.003	0.088	0.231

**Table 4:** Comparison of pain visual simulation scores between the two groups (VAS).

Observation index	Group	*n*	1 week after surgery	4 weeks after surgery	12 weeks after surgery
VAS (scores)	Control group	36	2.50 ± 0.64	1.68 ± 0.41	1.10 ± 0.29
	Observation group	24	4.33 ± 0.80	2.93 ± 0.195	1.49 ± 0.42
*χ* ^2^/*t*			9.366	10.168	3.847
*P*			0.000	0.000	0.000

**Table 5:** Quality of life scores in both groups.

Projects	1 week before surgery		1 week after surgery		12 weeks after surgery	
	Observation group (*n* = 24)	Control group (*n* = 36)	Observation group (*n* = 24)	Control group (*n* = 36)	Observation group (*n* = 24)	Control group (*n* = 36)
*QLQ-C30 functional dimensions*						
Physical function	88.75 ± 9.94	87.28 ± 11.51	71.29 ± 11.99	57.37 ± 8.44^∗^	78.29 ± 9.37	65.25 ± 8.17^∗^
Integrated quality of life	72.63 ± 8.14	69.14 ± 8.28	59.25 ± 4.43	45.47 ± 5.17^∗^	65.13 ± 4.61	55.44 ± 4.27^∗^
*QLQ-C30 symptom dimension*						
Fatigue	23.17 ± 5.80	24.79 ± 4.26	52.46 ± 6.28	68.97 ± 4.97^∗^	40.08 ± 5.17	57.67 ± 4.22^∗^
Pain	15.67 ± 5.62	17.08 ± 4.42	45.50 ± 8.45	62.53 ± 8.70^∗^	25.04 ± 6.64	40.36 ± 10.35^∗^
*QLQ–STO22 symptom dimension*						
Difficulty swallowing	39.75 ± 7.55	41.25 ± 8.23	20.04 ± 4.72	21.47 ± 5.78	11.79 ± 3.05	11.86 ± 3.93
Stomach pain	20.33 ± 7.9	19.22 ± 5.87	28.92 ± 6.37	31.25 ± 6.98	37.5 ± 6.24	38.06 ± 6.51

^∗^ *P* < 0.05 was found to be significant.

**Table 6:** Comparison of postoperative follow-up between the two groups (*n*, (%)).

Group	*n*	Death	Transfer of recurrence	Eat well	Normal defecation	Reverse acid	Nausea and vomiting	Edge of pain
Control group	36	3 (8.33)	5 (13.89)	15 (41.67)	30 (83.33)	15 (41.67)	5 (13.89)	16 (44.44)
Observation group	24	2 (8.33)	3 (12.50)	19 (79.17)	18 (75.00)	3 (12.50)	4 (16.67)	4 (16.67)
*χ* ^2^/*t*/*Z*		0.227	0.024	8.247	0.625	5.833	0.087	5.000
*P*		0.634	0.877	0.004	0.429	0.015	0.768	0.025

## Data Availability

The authors confirm that the data supporting the findings of this study are available within the article.
